This article has been retracted.

# *NLRC4* Gene Single Nucleotide Polymorphisms Are Associated with the Prognosis of Hemophagocytic Lymphohistiocytosis

**DOI:** 10.1155/2021/8581746

**Published:** 2021-12-10

**Authors:** Yan Li, Chengdong Sun, Liying Cui, Qiuying Wang

**Affiliations:** ^1^Department of Hematology, Xuanwu Hospital, Capital Medical University, Beijing 100053, China; ^2^Department of Infectious Diseases, Beijing Jishuitan Hospital, Beijing 100096, China

## Abstract

**Objective:**

To analyze and study the correlation between NLR family CARD domain-containing 4 (NLRC4) gene single nucleotide polymorphisms and the prognosis of patients with hemophagocytic lymphohistiocytosis (HLH).

**Methods:**

In this study, we retrospectively studied the clinical data of 62 HLH patients, including 40 males and 22 females. The genomic DNA was extracted, and the genotypes at rs385076 locus and rs479333 locus of the *NLRC4* gene were analyzed. The level of blood interleukin-18 (IL-18) was analyzed by enzyme-linked immunosorbent assay (ELISA).

**Results:**

Compared with the TT genotype at the *NLRC4* gene rs385076 locus, the mortality of HLH patients with TC genotype and CC genotype was higher (RR = 3.205, 95% CI: 1.277-4.788, *p* = 0.012; RR = 3.052, 95% CI: 1.098-4.753, *p* = 0.031). Taking the CC genotype at rs479333 of the *NLRC4* gene as a reference, HLH patients with CG genotype and GG genotype had a higher risk of death (RR = 3.475, 95% CI: 1.488-5.775, *p* = 0.003; RR = 2.986, 95% CI: 1.014-5.570, *p* = 0.047). *NLRC4* gene rs385076 T>C and rs479333 C>G were significantly related to the poor prognosis of HLH patients. The area under the curve (AUC) of the receiver operating curve (ROC) for the prognostic outcome of HLH with serum IL-18 level was 0.6813 (95% CI: 0.5365-0.8260, *p* = 0.0189). *NLRC4* gene rs385076 T>C and rs479333 C>G were related to higher serum IL-18 levels.

**Conclusion:**

*NLRC4* gene rs385076 T>C and rs479333 C>G are related to the poor prognosis of HLH patients.

## 1. Introduction

Hemophagocytic syndrome, also known as hemophagocytic lymphohistiocytosis (HLH), is due to the excessive activation and proliferation of macrophages, accompanied by decreased activities of natural killer (NK) cells and cytotoxic T lymphocytes (CTL), granzyme-dependent cytotoxicity defect, which in turn induce a series of clinical syndromes caused by immune dysfunction [1–3].

According to the different triggering factors of HLH, HLH includes primary HLH and secondary HLH. Primary HLH occurs mostly in children and adolescents, but rarely in adults. Secondary HLH is mostly caused by infections, tumors, and immune diseases. Recent studies have shown that the dysfunction of CTL, NK cells, and macrophages and the sharp increase in cytokine levels play an important role in the pathogenesis of HLH [4]. The continuous attention of research has led us to discover that more and more gene mutations are involved in the occurrence of HLH. For example, a meta-analysis result of 391 HLH patients and 975 controls showed that the *PRF1* Ala91Val polymorphism was related to the occurrence of HLH [5]. The study of Yang et al. [6] proved for the first time that the polymorphism of *STXBP2* rs2303116 was related to the pathogenesis of HLH. The above gene mutations affect the synthesis, transportation, anchoring, initiation, or membrane fusion of cytotoxic particles, resulting in the inability of cytotoxic particles to be secreted outside the cell; as a result, the killing function of CTL and NK cells is impaired, the target cells cannot be eliminated, and they participate in the pathogenesis of primary HLH.

The *NLRC4* gene is located on the human 2p22.3 chromosome; NLRC4 is a multiprotein complex whose activation is related to the secretion of inflammatory factors [7, 8]. Studies have shown that NLRC4 inflammasome can release IL-1*β* and IL-18 to promote inflammation [9, 10]. Mutations in the *NLRC4* gene are related to the impaired immune regulation of macrophages; the gene mutation not only activates macrophages to produce IL-1*β* and IL-18, but also activates macrophage caspase-1, causing macrophages to phagocytose target cells and then apoptotic, reducing the number of functional macrophages [7, 11]. According to research, rs385076 and rs479333 gene polymorphisms were related to the occurrence of many diseases [12, 13]. The results of a meta-analysis showed that serum IL-18 levels were significantly increased both in primary HLH and secondary HLH [14]. Studies have confirmed that IL-18 plays an important role in the occurrence of HLH, and inhibiting IL-18 may be an effective strategy for the treatment of HLH [15]. Studies have shown that IL-18 plays a very important role in the pathogenesis of macrophage activation syndrome; in children with NLRC4 mutations, researchers have found that IL-18 circulates in the range of tens of nanograms/mL [16].

In this study, we explored the correlation between the single nucleotide polymorphisms of the *NLRC4* gene and the prognosis of HLH patients, aiming to provide valuable markers for the prognosis of HLH patients.

## 2. Materials and Methods

### 2.1. Subject

We retrospectively analyzed the clinical data of 62 HLH patients from 2018 to 2021, and the stored plasma samples were extracted; the patient's 1-year follow-up outcome information was collected. Among them, 40 were males and 22 were females, aged 25-84 years old. All patients had different degrees of fever and hepatomegaly, with heat duration of 2-8 weeks, 25 cases of splenomegaly, 18 cases of lymphadenopathy, 19 cases of skin and mucosal hemorrhage, and 8 cases of jaundice. The diagnosis of HLH conforms to the HLH 2004 diagnostic criteria [17].

### 2.2. Inclusion Criteria and Exclusion Criteria

Inclusion criteria were as follows. (1) Clinical data and laboratory test result data were available. (2) One-year follow-up outcome data was available. (3) Age ≥ 18 years. (4) A series of routine laboratory tests were performed during the diagnosis of the patient. Exclusion criteria were as follows: (1) clinical data and laboratory test result data not available, (2) patients with heart disease of grade II or above (including grade II) identified according to the New York Heart Association (NYHA) score, (3) HIV-infected patients, (4) patients with severe renal dysfunction (GFR < 15 mL/min), (5) patients with severe cirrhosis (MELD score > 20), (6) infection that cannot be controlled (including lung infection and intestinal infection), (7) severe mental illness, (8) a history of active tumor, (9) pregnant and lactating patients, (10) participating in other clinical researchers at the same time, and (11) persons with central nervous system involvement.

### 2.3. Gene Mutation Locus Selection and Analysis

The gene mutation sites we selected need to meet the following conditions. (1) Studies have reported that this mutation is pathogenic. (2) Based on the results of the 1000 Genomes Project database, the minor allele frequency (MAF) of this mutation site in the Chinese Han population > 0.05. (3) No studies have reported the correlation between this variant site and HLH. Sanger sequencing was used to analyze the genotypes at rs385076 and rs479333 of the *NLRC4* gene.

### 2.4. Laboratory Index Testing

We collected the results of patients' laboratory test indicators, including white blood cell (WBC) count, absolute number of neutrophils, platelets, hemoglobin, fibrinogen, lactate dehydrogenase (LDH), alanine aminotransferase (ALT), aspartate aminotransferase (AST), triglycerides (TG), total bilirubin (TBIL), prothrombin time (PT), activated partial thromboplastin time (APTT), albumin, and interleukin-18 (IL-18). WBC and PLT were detected by XE-5000 automatic five-category hematology analyzer (Sysmex, Japan). PT and APTT were detected by an automatic coagulation analyzer (Sysmex, Japan). The level of IL-18 was detected by enzyme-linked immunosorbent assay (ELISA). The levels of ALT, AST, TG, TBIL, LDH, hemoglobin, albumin, and fibrinogen were detected with a 7600X020 automatic biochemical analyzer (Hitachi, Japan).

### 2.5. Statistical Analysis

In this study, GraphPad prism (version 8.4.0, for Mac OS, San Diego, California, USA) was used for statistical analysis. Continuous data was expressed as mean ± standard deviation, and *t*-test was used for comparison and analysis between groups. Categorical data was expressed by *n* (%), and the *χ*^2^ test was used for the analysis between groups. Logistic regression analysis was used to study the correlation between *NLRC4* gene rs385076 and rs479333 single nucleotide polymorphisms and the relative risk (RR) of HLH. Age, gender, BMI, history of hypertension, history of diabetes, history of coronary heart disease, and EBV infection rate were used as covariates to calculate relative risk (RR) and 95% confidence interval (95% CI). The Kaplan-Meier method was used to analyze the differences in the prognostic outcomes of HLH patients with different genotypes. All tests were two-tailed, and *p* < 0.05 indicated that the difference was statistically significant.

## 3. Results

### 3.1. Clinical Data

The clinical data of 62 HLH patients selected in this study are shown in Table 1. They were 25-84 years old, with an average of 59.68 ± 11.33 years old. Among them, 40 cases were male, accounting for 64.52%, and 22 cases were female, accounting for 35.48%. Follow-up results showed that 22 cases died and 40 cases survived. The analysis results showed that there were no significant differences in age, gender, and body mass index (BMI) between the death group and the survival group of HLH patients (*p* > 0.05). The proportion of hypertension, diabetes, coronary heart disease, and EBV infection rate of HLH patients in the death group was significantly higher than that of HLH patients in the survival group, and the differences were statistically significant (*p* < 0.05).

### 3.2. Laboratory Testing Indicators

The laboratory index test results of HLH patients are shown in Table 2. The analysis results showed that there were no significant differences between the death group and the survival group in the WBC, absolute number of neutrophils, hemoglobin, fibrinogen, LDH, ALT, TG, TBIL, PT, and APTT (*p* > 0.05), while the platelet and albumin levels of HLH patients in the death group were significantly lower than those of the survival group, the AST level was significantly higher than that of the survival group, and the differences were statistically significant (*p* < 0.05).

### 3.3. Analysis of Single Nucleotide Polymorphism of the *NLRC4* Gene

The genotypes and allele frequencies of *NLRC4* rs385076 and rs479333 in HLH patients of the death group and the survival group are shown in Table 3. Compared with the TT genotype at the *NLRC4* rs385076 locus, after adjusting for the age, gender, BMI, history of hypertension, diabetes, coronary heart disease, and history of EBV infection in HLH patients, the TC genotype (RR = 3.205, 95% CI: 1.277-4.788, *p* = 0.012) and CC genotype (RR = 3.052, 95% CI: 1.098-4.753, *p* = 0.031) of HLH patients had a higher mortality rate. The risk of death of HLH patients under the dominant model was significantly increased (RR = 3.133, 95% CI: 1.543-5.029, *p* < 0.001), but the risk of death in HLH patients in the recessive model did not change significantly (RR = 2.311, 95% CI: 0.882-3.393, *p* = 0.091). From the perspective of alleles, it was found that the death risk of HLH carrying the C allele at rs385076 was 2.262 times that of the T allele carriers (95% CI: 1.359-3.347, *p* = 0.002).

Taking the CC genotype at rs479333 of the *NLRC4* gene as a reference, after adjusting the age, gender, BMI, history of hypertension, diabetes, coronary heart disease, and history of EBV infection, HLH patients with CG genotype and GG genotype had a higher risk of death (RR = 3.475, 95% CI: 1.488-5.775, *p* = 0.003; RR = 2.986, 95% CI: 1.014-5.570, *p* = 0.047). The risk of death of HLH patients under the dominant model was significantly increased (RR = 3.269, 95% CI: 1.580-6.092, *p* = 0.001), but the risk of death in HLH patients in the recessive model did not change significantly (RR = 1.985, 95% CI: 0.741-3.250, *p* = 0.188). From the perspective of alleles, G allele was a risk factor for death in HLH patients (RR = 2.487, 95% CI: 1.518-3.607, *p* < 0.012).

### 3.4. Single Nucleotide Polymorphisms of the *NLRC4* Gene and Prognostic Outcomes of HLH Patients

The prognostic outcomes of HLH patients with different genotypes at rs385076 and rs479333 of the *NLRC4* gene are shown in Figure 1. The analysis results showed that the prognostic outcomes of HLH patients with TT, TC, and CC genotypes at rs385076 of the *NLRC4* gene (Figure 1(a)) and the prognostic outcomes of HLH patients with CC, CG, and GG genotypes at rs479333 (Figure 1(b)) were significantly different (*p* < 0.01). Overall, rs385076 T>C and rs479333 C>G were significantly related to the poor prognosis of HLH patients.

### 3.5. IL-18 Level and Prognostic Outcome of HLH Patients

Our analysis showed that the serum IL-18 level of HLH patients in the survival group was significantly lower than that of HLH patients in the death group, and the difference was statistically significant (*p* = 0.006, Figure 2(a)). In addition, the receiver operating curve (ROC) was used to analyze the evaluation value of blood IL-18 level in the prognostic outcome of HLH, and the results showed that the area under the curve (AUC) was 0.6813 (95% CI: 0.5365-0.8260, *p* = 0.0189), the cut-off value is 45.75 ng/L, and the corresponding sensitivity and specificity are 59.09% and 80.00%, respectively. This result showed that blood IL-18 had a significant value in the prognosis assessment of HLH patients.

### 3.6. Single Nucleotide Polymorphism of the *NLRC4* Gene and Serum IL-18 Level

The serum IL-18 levels of HLH patients with different genes at the rs385076 locus and rs479333 locus of the *NLRC4* gene were analyzed, and the results are shown in Figure 3. The analysis results showed that rs385076 T>C and rs479333 C>G were related to higher serum IL-18 levels (Figures 3(a) and 3(b)).

## 4. Discussion

In this study, we retrospectively analyzed 62 HLH patients with *NLRC4* gene rs385076 locus and rs479333 locus single nucleotide polymorphisms and the prognostic outcome of HLH patients. We found that *NLRC4* gene rs385076 T>C and rs479333 C>G were associated with poor prognostic outcomes in HLH patients.

The clinical features of HLH include fever; enlarged liver, spleen, and lymph nodes; decreased peripheral blood cells; abnormal liver function; coagulopathy; and hemophilic cells in the bone marrow [18, 19]. However, due to the many triggering factors of HLH, its diagnosis still faces great difficulties [20]. Although the mortality rate of HLH has improved significantly in recent years, the mortality rate of HLH patients is still relatively high for both adults and children; the mortality rate of adult patients is as high as 22%-59% [21–23]. According to the results of research on HLH, the inflammatory factor storm caused by uncontrolled proliferation and expansion of immune system participants such as macrophages and T cells is one of the reasons for the higher mortality of HLH patients. In order to further increase the understanding of HLH, it is necessary to further explore the mechanisms related to the occurrence of HLH.

Since the perforin 1 gene defect was found to be associated with familial HLH in 1999, mutations in multiple genes associated with perforin have been found to be associated with familial HLH. HLH is a highly inflammatory disease. Studies have shown that there were a large number of inflammatory factors in HLH patients, including IL-1*β*, IL-2, IL-6, IL-8, TNF-*α*, and IFN-*γ*, and the higher the level of these cytokines, the worse the prognosis of HLH patients [24, 25].

The protein encoded by the *NLRC4* gene plays an important role in dealing with foreign pathogens, tissue damage, and innate immune response [26, 27]. NLRC4 inflammasome is activated after pathogen invasion is discovered and induces the large expression of IL-18 and IL-1*β*, leading to cell death, and it has also been proved that IL-18 and IL-1*β* participate in the inflammation induced by NLRC4 mutation in mouse models [10]. In fact, *NLRC4* gene mutations are related to the occurrence of a variety of autoinflammatory diseases, including autoinflammatory syndrome induced by cold [28], infant enteritis, and macrophage activation syndrome [29, 30]. One of the characteristics of the disease caused by NLRC4 mutation is the high level of serum IL-18; targeted inhibition of IL-18 may be a promising treatment option for the treatment of macrophage activation syndrome caused by NLRC4 mutation [31].

In this study, we found that compared with the TT genotype at the rs385076 locus of the *NLRC4* gene, the mortality of HLH patients with TC genotype and CC genotype was higher. Taking the CC genotype at rs479333 of the *NLRC4* gene as a reference, HLH patients with CG genotype and GG genotype had a higher risk of death. It prompts us that the *NLRC4* gene rs385076 T>C and rs479333 C>G are significantly related to the poor prognosis of HLH patients. Both rs385076 and rs479333 are located on the introns of *NLRC4* gene. Mutations do not affect the nucleotide sequence of the gene. However, these two SNP sites may be in the gene expression regulatory region, because both are related to the expression level of NLRC4 [13, 32]; however, we were unable to collect the expression data of NLRC4 and failed to confirm this hypothesis.

According to research, the rs385076 T allele was associated with lower IL-18 concentration and was a protective factor for cardiovascular-related death risk [11, 32]. The rs479333 G>C variant reduced the expression level of NLRC4, eventually leading to a decrease in IL-18 expression level [13]. Our research results showed that serum IL-18 levels were significantly related to the prognostic outcome of HLH patients and had certain value in diagnosing the poor prognostic outcome of HLH patients. IL-18 is a proinflammatory cytokine that can induce the polarization of Th1 and Th2 and promote various innate immune processes [33–35]. Recent studies have shown that macrophage abnormalities caused by NLRC4 inflammasome mutations are related to autoinflammation and macrophage activation syndrome [36]. The role of IL-18 in HLH may be mediated by its induction of IFN-*γ* and proinflammatory cytokines [37, 38]. In addition, studies had shown that IL-18 levels in patients with macrophage activation syndrome were significantly increased, and severe experimental macrophage activation syndrome had been found in IL-18 transgenic mice [39]. This proves the importance of free IL-18 for macrophage activation syndrome. Therefore, we speculate that the correlation between the *NLRC4* genes rs385076 T>C and rs479333 C>G and the poor prognosis of HLH patients may be mediated by IL-18.

Some deficiencies limit the value of our research. First of all, this is a retrospective study, limited by the size of the sample; we cannot ignore the limitations brought about by the small sample, and it needs to be further verified in a large sample. Secondly, we lack in vitro and in vivo experiments to further confirm our speculation, and further research is needed.

## 5. Conclusion

The *NLRC4* gene rs385076 T>C and rs479333 C>G are associated with elevated serum IL-18 expression levels and poor prognosis of HLH patients. The specific mechanism needs to be further verified in in vitro and in vivo models. The results of this study have certain guiding value for improving the poor prognosis of HLH patients.

## Figures and Tables

**Figure 1:** The prognostic outcome of HLH patients with different genotypes at rs385076 and rs479333 in the *NLRC4* gene. (a) Comparison of the prognostic outcomes of *NLRC4* gene rs385076 TT, TC, and CC genotypes. (b) Comparison of prognostic outcomes of *NLRC4* gene rs479333 CC, CG, and GG genotypes.

**Figure 2:** Blood IL-18 levels in HLH patients. (a) Comparison of serum IL-18 levels between HLH patients in the survival group and HLH patients in the death group. (b) The receiver operating curve (ROC) of serum IL-18 level to evaluate the prognostic outcome of HLH patients.

**Figure 3:** Single nucleotide polymorphism of the *NLRC4* gene and serum IL-18 level. (a) The comparison of serum IL-18 level between HLH patients with rs385076 TT, TC, and CC genotypes. (b) The comparison of serum IL-18 levels in HLH patients with rs479333 CC, CG, and GG genotypes.

**Table 1:** Clinical data.

Index	HLH (*n* = 62)	Death group (*n* = 22)	Survival group (*n* = 40)	*p*
Age	59.68 ± 11.33	58.68 ± 8.86	60.23 ± 12.56	0.612
Gender				
Male	40 (64.52%)	13 (59.09%)	27 (67.50%)	0.508
Female	22 (35.48%)	9 (40.91%)	13 (32.50%)	
BMI (kg/m^2^)	26.86 ± 2.94	27.02 ± 2.72	26.77 ± 3.09	0.752
History of hypertension [*n* (%)]				
Yes	23 (37.10%)	12 (54.55%)	11 (27.50%)	0.035
No	39 (62.90%)	10 (45.45%)	29 (72.50%)	
History of diabetes [*n* (%)]				
Yes	11 (17.74%)	8 (36.36%)	3 (7.50%)	0.004
No	51 (82.26%)	14 (63.64%)	37 (92.50%)	
History of coronary heart disease [*n* (%)]				
Yes	14 (22.58%)	10 (45.45%)	4 (10.00%)	0.001
No	48 (77.42%)	12 (54.55%)	36 (90.00%)	
EBV infection [*n* (%)]				
Yes	12 (19.35%)	8 (36.36%)	4 (10.00%)	0.012
No	50 (80.65%)	14 (63.64%)	36 (90.00%)	

HLH: hemophagocytic lymphohistiocytosis; BMI: body mass index; EBV: Epstein-Barr virus.

**Table 2:** Comparison of laboratory test indicators between the survival group and the death group of HLH patients (mean ± SD).

Index	Death group (*n* = 22)	Survival group (*n* = 40)	*t*	*p*
WBC (×10^9^/L)	2.49 ± 1.91	3.19 ± 1.39	1.657	0.103
Absolute number of neutrophils (×10^9^/L)	0.56 ± 0.24	0.53 ± 0.27	0.435	0.665
Platelets (×10^9^/L)	25.06 ± 12.00	64.70 ± 27.04	7.956	<0.001
Hemoglobin (g/L)	93.48 ± 46.29	95.26 ± 55.78	0.127	0.899
Fibrinogen (g/L)	1.49 ± 0.54	1.77 ± 0.74	1.559	0.124
LDH (U/L)	1259.59 ± 635.58	1007.01 ± 403.98	1.686	0.102
ALT (U/L)	224.78 ± 74.23	196.32 ± 71.74	1.476	0.145
AST (U/L)	311.04 ± 116.32	238.08 ± 94.37	2.679	0.010
TG (mmol/L)	3.03 ± 1.34	3.67 ± 1.84	1.434	0.157
TBIL (mmol/L)	54.48 ± 29.75	43.91 ± 15.36	1.556	0.131
PT (s)	15.32 ± 8.42	13.78 ± 7.01	0.770	0.444
APTT (s)	51.95 ± 13.61	48.50 ± 17.57	0.798	0.428
Albumin (g/L)	28.68 ± 6.44	45.88 ± 17.91	5.465	<0.001

HLH: hemophagocytic lymphohistiocytosis; WBC: white blood cells; LDH: lactate dehydrogenase; ALT: alanine aminotransferase; AST: aspartate aminotransferase; TG: triglyceride; TBIL: total bilirubin; PT: prothrombin time; APTT: activated partial thromboplastin time.

**Table 3:** Comparison of genotypes and allele frequencies at rs385076 locus and rs479333 locus of the *NLRC4* gene in the death group and the survival group of HLH patients.

	Death (*n* = 22)	Survive (*n* = 40)	RR (95% CI)^#^	*p*
rs385076				
Genotype				
TT	11 (50.00%)	36 (90.00%)	1.00 (reference)	
TC	6 (27.27%)	2 (5.00%)	3.205 (1.277-4.788)	0.012
CC	5 (22.73%)	2 (5.00%)	3.052 (1.098-4.753)	0.031
Dominant model			3.133 (1.543-5.029)	0.001
Recessive model			2.311 (0.882-3.393)	0.091
Allele				
T	27 (61.36%)	70 (87.50%)	1.00 (reference)	
C	17 (38.64%)	10 (12.50%)	2.262 (1.359-3.347)	0.002
rs479333				
Genotype				
CC	9 (40.91%)	34 (85.00%)	1.00 (reference)	
CG	8 (36.36%)	3 (7.50%)	3.475 (1.488-5.775)	0.003
GG	5 (22.73%)	3 (7.50%)	2.986 (1.014-5.570)	0.047
Dominant model			3.269 (1.580-6.092)	0.001
Recessive model			1.985 (0.741-3.250)	0.188
Allele				
C	26 (59.09%)	71 (88.75%)	1.00 (reference)	
G	18 (40.91%)	9 (11.25%)	2.487 (1.518-3.607)	<0.001

RR: relative risk; CI: confidence interval. ^#^Adjusted the age, gender, BMI, history of hypertension, diabetes, coronary heart disease, and EBV infection of HLH patients.

## Data Availability

The data in this study can be obtained from the corresponding author with appropriate reasons.
